The article "Establishment and Validation of an MTORC1 Signaling-Related Gene Signature to Predict Overall Survival in Patients with Hepatocellular Carcinoma" was retracted in 2024. Reasons: signs of a paper mill; suspected computer-generated content; unreliable results or conclusions; concerns about the data.

# Establishment and Validation of an MTORC1 Signaling-Related Gene Signature to Predict Overall Survival in Patients with Hepatocellular Carcinoma

**DOI:** 10.1155/2021/6299472

**Published:** 2021-11-22

**Authors:** Zheng Yao, Song Wen, Jun Luo, Weiyuan Hao, Weiren Liang, Yutang Chen

**Affiliations:** Department of Radiology Intervention, Cancer Hospital of the University of Chinese Academy of Sciences (Zhejiang Cancer Hospital), Hangzhou, 310000 Zhejiang, China

## Abstract

**Background:**

Accurate and effective biomarkers for the prognosis of patients with hepatocellular carcinoma (HCC) are poorly identified. A network-based gene signature may serve as a valuable biomarker to improve the accuracy of risk discrimination in patients.

**Methods:**

The expression levels of cancer hallmarks were determined by Cox regression analysis. Various bioinformatic methods, such as GSEA, WGCNA, and LASSO, and statistical approaches were applied to generate an MTORC1 signaling-related gene signature (MSRS). Moreover, a decision tree and nomogram were constructed to aid in the quantification of risk levels for each HCC patient.

**Results:**

Active MTORC1 signaling was found to be the most vital predictor of overall survival in HCC patients in the training cohort. MSRS was established and proved to hold the capacity to stratify HCC patients with poor outcomes in two validated datasets. Analysis of the patient MSRS levels and patient survival data suggested that the MSRS can be a valuable risk factor in two validated datasets and the integrated cohort. Finally, we constructed a decision tree which allowed to distinguish subclasses of patients at high risk and a nomogram which could accurately predict the survival of individuals.

**Conclusions:**

The present study may contribute to the improvement of current prognostic systems for patients with HCC.

## 1. Introduction

Hepatocellular carcinoma (HCC) is the most common form of liver cancer globally and is a leading cause of cancer-related mortality [1, 2]. Currently, the available potentially curative approaches are only suitable for early-stage HCC cases [3], whereas the majority of HCC patients are diagnosed at relatively advanced stages and thus have poor prognosis [1, 4]. Additionally, biomarkers, as emerging tools, play a pivotal role in the diagnosis, prognosis, and prediction of treatment responses, leading to the improvement of patient stratification and clinical outcomes [5]. However, accurate and sufficient biomarkers are still lacking; therefore, there is an urgent need to tackle this limitation by identifying network-based biomarkers for the discrimination of HCC patients with unfavorable outcomes.

The article "Establishment and Validation of an MTORC1 Signaling-Related Gene Signature to Predict Overall Survival in Patients with Hepatocellular Carcinoma" was retracted in 2024. Reasons: signs of a paper mill; suspected computer-generated content; unreliable results or conclusions; concerns about the data.

MTORC1 signaling belongs to the mTOR pathway, which also includes MTORC2 signaling [6]. It has been proved that aberrant activation of MTORC1 signaling results in tumorigenesis and cancer progression through enhanced cell survival and metastasis [7, 8]. Various research groups have reported that the expression levels of components or modulators of MTORC1 signaling, such as p-AKT and RICTOR, are associated with poor survival in patients with HCC [9]. A recent study reported that a six-gene signature based on MTORC1 signaling can be used for the prognosis of patients with HCC [10]. Nevertheless, a systematic MTORC1 signaling signature based on this coexpression network has yet to be constructed for the application to HCC risk stratification.

In the present study, we found that active MTORC1 signaling was the most predominant predictor of overall survival among a variety of cancer hallmarks. Moreover, by applying multiple bioinformatic approaches, an MTORC1 signaling-related gene signature (MSRS) was created; this was found to be robust for risk discrimination via validation in different cohorts. Furthermore, a decision tree and nomogram that integrated multiple clinical parameters were generated to optimize the entire procedure of risk stratification for HCC patients.

## 2. Material and Methods

### 2.1. Data Processing

The clinicopathological details and survival data of the training dataset GSE14520 [11] and the validation dataset I GSE76427 [12] were downloaded from the GEO database (http://www.ncbi.nlm.nih.gov/geo/). The same information for the validation cohort II TCGA-LIHC [13] was derived from https://portal.gdc.cancer.gov/projects/TCGA-LIHC. All data used in this study were normalized.

### 2.2. Pathway Enrichment and Construction of an MTORC1 Signaling-Related Signature

The R package “survival” was applied to perform Cox regression analysis for the assessment of the expression levels of hallmark gene sets [14, 15]. Single-sample gene set enrichment analysis (ssGSEA) scores for each hallmark were determined using the R package “gsva.” The construction of a scale-independent coexpression network and module was carried out using the “WGCNA” R package [16]. After the identification of the black module as the one most enriched in genes representing the MTORC1 gene signature, least absolute shrinkage and selection operator (LASSO) Cox regression analysis was conducted to select the most relevant genes [17]. Finally, an MTORC1 signaling-related signature (MSRS) was constructed by calculating the gene expression levels with the corresponding LASSO Cox coefficients as previously described [18].

### 2.3. Bioinformatic Analysis

SPSS Statistics (IBM version 20), GraphPad Prism (version 7.0), Stata (version 12), and R software (version 4.1.1,http://www.r-project.org) were used to perform GSEA [19, 20] and generate the plots. The *Z*-score that is used to estimate the “enrichment” of the entire gene set was applied to calibrate ssGSEA scores [21] and MSRS, and the Kaplan–Meier approach was used to construct patient survival plots. Quantification of predictive power in terms of time-dependent receiver operating characteristic [22] was carried out using the R package “survival-ROC” [23]. A decision tree was generated by recursive partitioning analysis using the R package “rpart” [24]. A nomogram and a correlation curve were constructed using the R package “rms” [25]. Codes for all the algorithms used in this study can be obtained by request to the corresponding author.

The article "Establishment and Validation of an MTORC1 Signaling-Related Gene Signature to Predict Overall Survival in Patients with Hepatocellular Carcinoma" was retracted in 2024. Reasons: signs of a paper mill; suspected computer-generated content; unreliable results or conclusions; concerns about the data.

### 2.4. Statistical Analysis

The log-rank test was used to evaluate differences between the survival of two patient groups. Student's *t*-test or one-way analysis of variance (ANOVA) was used to determine statistically significant differences between the indicated groups. *p* < 0.05 was considered as threshold for statistical significance. ^∗^, 0.01 < *p* < 0.05; ^∗∗^, 0.001 < *p* < 0.01; ^∗∗∗^, 0.0001 < *p* < 0.001; ^∗∗∗∗^*p* < 0.0001; ns: not significant.

## 3. Results

### 3.1. Enriched Expression of MTORC1 Signaling Components Is a Primary Risk Factor for the Survival of Patients with HCC

To identify pathways or cellular processes suitable as novel primary factors for survival prediction in patients with HCC, we calculated the ssGSEA score of each hallmark from the Molecular Signatures Database (MSigDB) in the training cohort GSE14520, which includes transcriptomic data from 221 HCC patients. After ranking the hallmarks according to their Cox coefficients, we observed that MTORC1 signaling was significantly overrepresented with respect to other pathways or processes, including angiogenesis, KRAS signaling, and UV response, thereby becoming the most significant primary factor for predicting the overall survival of patients with HCC (Figure 1(a)). As shown in Figure 1(b), the ssGSEA *Z*-scores of genes implied in MTORC1 signaling were increased in deceased patients compared to those in patients who were alive during follow-up. Moreover, patient survival was significantly reduced (HR = 2.207, *p* = 0.00019) in patient subgroups exhibiting higher ssGSEA scores for MTORC1 signaling-related genes. Collectively, these results suggest that MTORC1 signaling is a promising primary factor for overall survival prediction in patients with HCC.

### 3.2. Construction of an MTORC1 Signaling-Related Signature to Predict the Outcome of HCC Patients

Next, we aimed to establish a robust MTORC1 signaling-related signature (MSRS) to better predict the survival outcome of patients with HCC. First, we performed sample clustering on the training dataset, and three samples (above the threshold indicated by the red line) were excluded as outliers in order to carry out more accurate further analysis (Figure 2(a)). After selecting power 5 as the optimal threshold for the scale-independent coexpression network (Figure 2(b)), we carried out weighted gene coexpression network analysis (WGCNA). This pointed at the black module (*r* = 0.6, *p* = 4*e*^−23^) as the module most correlated with MTORC1 signaling (Figures 2(c) and 2(d)). Furthermore, we performed univariate Cox regression analysis using isolated hub genes (with a *p* value for gene significance < 0.0001) as the input. As a result, 11 candidate markers (six positive and five negative) were identified as the most correlated with MTORC1 signaling (Figure 2(e)). As the tuberous sclerosis (TSC) complex is one of the most crucial negative regulators of MTORC1 signaling [26], we examined the correlations between the expression of *TSC2*, encoding a component of the TSC complex, and that of the 11 identified key hub genes. As expected, we observed strong reverse correlations between the expression levels of *TSC2* and those of risk genes such as *CALU* and positive correlations between *TSC2* expression and that of protective genes such as *CLN3* (Figure 2(f)).

The article "Establishment and Validation of an MTORC1 Signaling-Related Gene Signature to Predict Overall Survival in Patients with Hepatocellular Carcinoma" was retracted in 2024. Reasons: signs of a paper mill; suspected computer-generated content; unreliable results or conclusions; concerns about the data.

### 3.3. The MSRS Enables to Predict Poor Survival of Patients in the Training Dataset

We proceeded to investigate whether the MSRS is capable of representing the status of MTORC1 signaling. As expected, GSEA confirmed that the MSRS was significantly correlated with MTORC1 signaling activation in the MSRS-high subgroup (Figure 3(a)). In addition, similar to MTORC1 signaling (Figure 1(b)), the MSRS score was increased in live patients when compared with dead patients in the aforementioned training dataset (Figure 3(b)). Moreover, patient survival analysis showed that HCC patients with high MSRS scores had a poor prognosis (Figure 3(c)). Subsequently, we aimed to test the accuracy of diverse pathological parameters for predicting the overall survival of patients with HCC. Of note, tROC quantification revealed that among all the tested clinical variables, the MSRS was the best prognosis indicator in the training cohort (Figure 3(d)). In line with this result, multivariate Cox regression analysis suggested that the MSRS and TNM stage are two distinct risk factors significantly affecting overall survival (Figure 3(e)). Taken together, our results demonstrated that the MSRS may act as an independent risk factor for overall survival prognosis in patients with HCC.

The article "Establishment and Validation of an MTORC1 Signaling-Related Gene Signature to Predict Overall Survival in Patients with Hepatocellular Carcinoma" was retracted in 2024. Reasons: signs of a paper mill; suspected computer-generated content; unreliable results or conclusions; concerns about the data.

### 3.4. Validation of the MSRS as a Predicting Factor for Worse Prognosis in Two Additional Datasets

To further evaluate the prognostic robustness of the MSRS, we applied the methodology described above to two other datasets, GSE76427 (*N* = 115) and TCGA-LIHC (*N* = 369). Similar to the training cohort, the MSRS was significantly correlated with MTORC1 signaling in both datasets (Figures 4(a) and 4(d)). Moreover, MSRS scores were higher in deceased patients than in patients who were alive during follow-up (Figures 4(b) and 4(e)). Consistent with this data, survival analysis revealed that the outcomes of MSRS-high patients were worse than those of MSRS-low patients (Figures 4(c) and 4(f)). Since the second dataset consisted of a larger number of patients, we focused on the survival data from the first 6 years of this cohort to test the prediction robustness of the MSRS in relatively early stages of HCC. Interestingly, an even more significant difference between MSRS-high and MSRS-low patients was detected (Figure 4(g)). Furthermore, multivariate Cox regression modeling showed that the MSRS and TNM stage were independent predictors of overall survival in TCGA-LIHC cohort (Figure 4(h)). Therefore, we confirmed that the MSRS can be utilized in various cohorts as a highly effective survival predictor.

### 3.5. Effectiveness of the MSRS as a Prognostic Indicator of Worse Outcome in a Combined Cohort and Patient Subcategories

To obtain a better overview of the prognostic value of the MSRS, we combined the training cohort with the two validation cohorts and performed additional analysis including comprehensive clinicopathological information of patients. Notably, we found that the *Z*-scores of MSRS genes were significantly increased in patients who died within 3 years or between 3 and 6 years from symptom onset in comparison with those of live patients in the pooled cohort (Figure 5(a)). Moreover, the MSRS could also distinguish high-risk HCC patients from the whole population (Figure 5(b)) or within multiple subcategories, such as patients with late TNM stages (stages II–IV, Figure 5(c)), patients of different age groups (Figure 5(d)), and males but not females (Figure 5(e)). In conclusion, we demonstrated that the MSRS is a useful survival predictor in both the whole population and certain subgroups.

### 3.6. MSRS Analysis Increases the Accuracy of Risk Stratification and Survival Prediction when Combined with Clinical Parameters

To optimize the process of risk discrimination for overall survival, we generated a decision tree (Figure 6(a)). TNM stage and the MSRS, but not gender or age, were retained in the decision tree to predict the survival of patients who were finally grouped into three subclasses, that is, low risk, intermediate risk, and high risk (Figures 6(a) and 6(b)). Of note, the difference between patients with high and low risk was significant in terms of overall survival probabilities (Figure 6(c)). Moreover, multivariate Cox regression analysis indicated that both the MSRS and TNM stage were robust indicators of overall survival (Figure 6(d)). Ultimately, to determine the risk and predict the survival of patients with HCC, we constructed a nomogram by combining MSRS analysis with that of other valuable clinical parameters (Figure 6(e)). Interestingly, we observed a positive correlation between the predicted 5-year survival and the actual 5-year survival of individuals (Figure 6(f)), suggesting that the generated nomogram holds great potential to support risk assessment and survival prediction of HCC patients.

The article "Establishment and Validation of an MTORC1 Signaling-Related Gene Signature to Predict Overall Survival in Patients with Hepatocellular Carcinoma" was retracted in 2024. Reasons: signs of a paper mill; suspected computer-generated content; unreliable results or conclusions; concerns about the data.

## 4. Discussion

MTORC1 signaling is a pivotal pathway triggered by various environmental stimuli, such as growth factors, amino acids, and increased cellular energy levels [6, 8, 27]. As a downstream target of the AKT and RAS-ERK pathways, MTORC1 signaling contributes greatly to the regulation of cell survival and metabolism during cancer progression [28]. Notably, the proactivation of mTOR/MTORC1 signaling has been shown to be correlated with poor outcome in patients with breast cancer, bladder cancer, and HCC [29–32]. In particular, the expression of regulators or components of the MTORC1 or MTORC2 pathways, including p-AKT and RICTOR, is elevated in 40–50% of patients with HCC [33, 34]. Although previous studies have suggested a valuable role of MTORC1 signaling in discriminating high-risk HCC patients, only the expression levels of individual genes in the MTORC1 pathway or upstream modulators or downstream targets of MTORC1 signaling have been considered so far; these may not represent the exact status of this pathway. Hence, an MTORC1-related gene signature based on gene networks was required to optimize its application to the prognosis of HCC patients.

In the present study, MTORC1 signaling was found to be enriched in HCC patients and validated as a key primary risk factor for the overall survival of HCC patients by applying Cox regression analysis to the training dataset. Next, we carried out WGCNA for the selection of MTORC1-related gene modules and LASSO Cox regression analysis for the construction of an MSRS including the most robust candidate genes. Subsequently, the predictive value of the MSRS was validated in the training cohort, two validation cohorts, and in multiple subgroups of the pooled cohort; this strongly suggests that the MSRS can be applied as a reliable predictor for the prognosis of HCC patients. Finally, a decision tree was established to optimize risk discrimination by including information on TNM stages. Also, a nomogram was constructed to integrate the prognostic power of the MSRS with that of other clinical features, for more accurate risk prediction. To improve the research value in the future, we would like to check the importance of MTORC1 signaling using some HCC models such as *in vitro* genetic approaches or antagonists/agonists for manipulating MTORC1 signaling in HCC cell lines. Mouse model such as Diethylnitrosamine- (DEN-) induced HCC model [35] can also be applied to check the MTORC1 signaling activation in mice and validate the prognostic value of the MSRS.

The article "Establishment and Validation of an MTORC1 Signaling-Related Gene Signature to Predict Overall Survival in Patients with Hepatocellular Carcinoma" was retracted in 2024. Reasons: signs of a paper mill; suspected computer-generated content; unreliable results or conclusions; concerns about the data.

A recent study showed that an MTORC1 signaling signature involved in six genes was generated and could be utilized for the prognosis of HCC patients [10]. Although they performed analysis on RNA sequencing data from TCGA database, while we applied a diverse cohort, MOTRC1 signaling was enriched in both studies, indicating the prognostic significance of this pathway for patients with HCC. Furthermore, we established a decision tree which can better aid to the prognosis based on the MTORC1 signaling.

Although a few candidate genes have been investigated in multiple cancers, a large proportion of them are still poorly studied in the context of MTORC1 signaling regulation. For instance, phosphoglycerate kinase 1 (*PGK1*), a candidate predictor gene with a high coefficient, has been shown to serve as an indispensable enzyme in the aerobic glycolysis pathway and thus as a promoter of cancer cell survival and chemoradiotherapy resistance in cancer patients [36]. Conversely, enolase-1 (*ENO1*) promotes the invasion and metastasis of cancer cells by altering a variety of signaling pathways such as the PI3K/AKT pathway [37–39]. Considering the lack of data on the biological effects of the biomarkers included in our MSRS, further functional studies are required to verify the potential links between these and MTORC1 signaling, for a better understanding of their roles as MSRS components.

Moreover, although the constructed MSRS has been demonstrated to be a powerful risk predictor for patients with HCC, its prognostic value should be further tested and validated in cohorts including a larger number of patients; such prospective trials may support the clinical use of this promising novel predictor of HCC outcome.

## Figures and Tables

**Figure 1:** MTORC1 signaling is identified as a primary factor for the survival of patients with HCC. (a) Cox regression analysis for the identification of primary factors affecting the overall survival (OS) of HCC patients. (b) Single-sample gene set enrichment analysis (ssGSEA) scores of MTORC1 signaling in patients who were alive or dead during follow-up. (c) Kaplan–Meier plot indicating the survival probabilities of HCC patients stratified by their ssGSEA score of MTORC1 signaling.

The article "Establishment and Validation of an MTORC1 Signaling-Related Gene Signature to Predict Overall Survival in Patients with Hepatocellular Carcinoma" was retracted in 2024. Reasons: signs of a paper mill; suspected computer-generated content; unreliable results or conclusions; concerns about the data.

**Figure 2:** Construction of an MTORC1 signaling-related signature (MSRS). (a) Cluster analysis of the patients' gene expression data. (b) Plot showing scale-free topology (left) and mean connectivity (right). (c) Results of WGCNA of transcriptomic data and ssGSEA Z-scores of MTORC1 signaling genes. (d) Correlations between the modules (labeled with different colors) and MTORC1 signaling. The black module, displaying the highest correlation, is highlighted. (e) Plot indicating hub gene candidates derived from the black module. (f) Correlations between *TSC2* expression and that of genes belonging to the MSRS.

**Figure 3:** The MSRS enables to predict unfavorable outcome in the training dataset. (a) GSEA results confirming the prognostic robustness of the MSRS. (b) Comparison of MSRS scores between patients who were alive (*N* = 138) or dead (*N* = 85) during follow-up. (c) Kaplan–Meier plot indicating the survival probabilities of HCC patients stratified by their MSRS scores. (d) tROC assessment demonstrating the accuracy of the MSRS for predicting patient survival. (e) Multivariate Cox regression analysis for the validation of the MSRS as a risk factor.

**Figure 4:** Validation of the MSRS as a predicting factor for worse prognosis in two additional datasets. (a) GSEA results confirming the prognostic value of the MSRS in the GSE76427 dataset (*N* = 115). (b) Comparison of MSRS scores between patients of the GSE76427 dataset who were alive (*N* = 92) or dead (*N* = 23) during follow-up. (c) Kaplan–Meier plot indicating the survival probabilities of HCC patients of the GSE76427 dataset stratified by their MSRS scores. (d) GSEA results confirming the prognostic value of the MSRS in TCGA-LIHC dataset (*N* = 369). (e) Comparison of MSRS scores between patients of TCGA-LIHC dataset who were alive (*N* = 240) or dead (*N* = 129) during follow-up. (f) Kaplan–Meier plot indicating the survival probabilities of HCC patients of TCGA-LIHC dataset stratified by their MSRS scores. (g) Kaplan–Meier plot indicating the survival probabilities (<6 years) of HCC patients of TCGA-LIHC dataset stratified by their MSRS scores. (h) Multivariate Cox regression analysis for the validation of the MSRS as a risk factor in TCGA-LIHC dataset (only the parameters relative to the first 6 years were included).

**Figure 5:** The MSRS serves as a prognostic indicator for poor outcome in a combined cohort and subcategories. (a) Comparison of MSRS *Z*-scores in alive patients (*N* = 338), patients who died within 3 years (*N* = 160), and patients who died between 3 and 6 years (*N* = 33). (b–e) Kaplan–Meier plot indicating the survival probabilities, in terms of overall survival, of HCC patients stratified by their MSRS scores in the (b) whole population or distinguished according to (c) early (left) or (c) late (right) TNM stages, (d) age under 65 (left) or over (d) 65 (right), and (e) gender.

The article "Establishment and Validation of an MTORC1 Signaling-Related Gene Signature to Predict Overall Survival in Patients with Hepatocellular Carcinoma" was retracted in 2024. Reasons: signs of a paper mill; suspected computer-generated content; unreliable results or conclusions; concerns about the data.

**Figure 6:** MSRS analysis increases the accuracy of risk stratification and survival prediction when combined with clinical parameters. (a, b) Decision tree for improving the risk stratification process. (c) Kaplan–Meier plot indicating the quality of the decision tree in terms of risk prediction. (d) Multivariate Cox regression analysis demonstrating the significance of diverse variables as primary factors. (e) Nomogram for evaluating the risk for a single patient. (f) Correlation between the actual 5-year survival of patients and that predicted by the nomogram.

## Data Availability

The data used to support the findings of this study are included within the article.
